# Recognition of Badminton Shot Action Based on the Improved Hidden Markov Model

This article has been retracted.

**DOI:** 10.1155/2021/7892902

**Published:** 2021-10-07

**Authors:** Chao Ma, Dayang Yu, Hao Feng

**Affiliations:** ^1^Qinhuangdao Campus, Northeast Petroleum University, Daqing 163000, Heilongjiang, China; ^2^Department of Physical Education, Zibo Vocational Institute, Zibo 255000, Shandong, China; ^3^Police Physical Education Department, Hebei Vocational College For Correctional Police, Shijiazhuang 050081, Hebei, China

## Abstract

In recent years, with the rapid development of sports, the number of people playing various sports is increasing day by day. Among them, badminton has become one of the most popular sports because of the advantages of fewer restrictions on the field and ease of learning. This paper develops a wearable sports activity classification system for accurately recognizing badminton actions. A single acceleration sensor fixed on the end of the badminton racket handle is used to collect the data of the badminton action. The sliding window segmentation technique is used to extract the hitting signal. An improved hidden Markov model (HMM) is developed to identify standard 10 badminton strokes. These include services, forehand chop, backhand chop the goal, the forehand and backhand, forehand drive, backhand push the ball, forehand to pick, pick the ball backhand, and forehand. The experimental results show that the model designed can recognize ten standard strokes in real time. Compared with the traditional HMM, the average recognition rate of the improved HMM is improved by 7.3%. The comprehensive recognition rate of the final strokes can reach up to 95%. Therefore, this model can be used to improve the competitive level of badminton players.

## 1. Introduction

Badminton is an Olympic discipline, and it is one of the most popular racket sports worldwide. With the rapid growth of artificial intelligence, performance analysis in sports has undergone fundamental changes in recent years [1]. Generally, manual analysis performed by trained sport science experts has some drawbacks such as time-consuming, time-intensive, and subjective. Analysis for sports events is crucial to understanding the physical and technical demands related to sports performance. Sports action recognition systems are developed to perform analysis in sport science, provide objective measurement, and enhance the efficiency and accuracy of sports performance [2, 3]. Generally, sports action recognition systems are developed using machine and deep learning approaches with data measured by an inertial and magnetic sensor or by computer vision technologies [4].

Sports actions recorded by the camera can be applied for athlete's pose estimation and movement analysis [5]. The computer vision-based activity recognition system's processes, mainly dependent on the sport and camera type, involve player tracking, targeted motion recognition, and temporal cropping [6]. This approach can provide rapid analysis and real-time feedback for coaches and athletes. However, the computer vision-based action recognition system is limited to specific environments and requires more computing power. An alternative approach for sports action recognition is to use inertial sensors for data collection. The sensors are wearable and composed of gyroscopes, accelerometers, and magnetometers [7, 8]. Wearable devices with embedded inertial sensors are commonly used in various applications such as gait analysis, activity recognition healthcare, disease monitoring, and navigation [9].

Recently, several researchers have developed wearable sports activity recognition and monitoring systems, football, badminton, tennis, baseball, golf, basketball, table tennis, volleyball, etc. [10]. The wearable inertial sensors can measure linear and angular accelerations generated by gestures and motions during sports training and competitions [11]. The wearable inertial sensor-based activity recognition system benefits are low cost, light-weighted, small-sized, and require minimum power for operation. Generally, the sports action recognition process involves several signal processing procedures such as raw signal filtering, signal windowing, normalization, prominent feature extraction, feature reduction/selection, and classification actions [12]. For example, Margarito et al. [13] extracted eleven acceleration features from the thirteen most common time- and frequency-domain features using the relief method. For eight-action classification, they used naïve Bayes (NB), logistic regression (LR), decision tree (DT), and artificial neural network (ANN) classifiers. These activities included cross-trainer, cycling, rowing, squatting, stepping, running, weightlifting, and walking. Ermers et al. [14] combined the DT classifier with the ANN to classify activities such as sitting, lying down, standing, walking, rowing with a rowing machine, running, and cycling with an exercise bike. A Nordic walking, playing football, and cycling with a regular bike using the seven time- and frequency-domain features were extracted from the accelerometers and GPS sensor signals. Mitchell et al. [15] used a smartphone accelerometer and employed discrete wavelet transform- (DWT-) based support vector machines (SVMs) optimized by the minimal sequential optimization (SMO) algorithm to recognize the seven sports activities. Wang et al. [16] used gyroscope and accelerometer signals in combination followed by principal component analysis (PCA) to obtain three features from the twelve statistical features and three morphological features. These are input to the support vector machine (SVM) classifier for classifying elite, subelite, and amateur volleyball players.

Our literature review shows that many researchers in machine learning have focused on inertial-sensing-based sports activity classification. A wearable badminton activity recognition system is developed using the hidden Markov model (HMM) in this paper. The main contributions of this paper are as follows:

- This paper proposes a sports action recognition algorithm for badminton hitting action and implements a real-time recognition system for badminton actions.
- The system uses a single acceleration sensor fixed at the end of the badminton racket handle to collect action data. It uses sliding window data segmentation technology to extract hitting signals.
- An improved HMM training model is proposed to identify ten standard badminton shots and achieved the highest recognition accuracy of 95%.

The rest of the paper is organized as follows: Section 2 provides the background and related work. The proposed improved HMM is explained in Section 3. The results are illustrated in Section 4. The conclusion is given in Section 5. Finally, the limitation and future work are given in Section 6.

## 2. Background

### 2.1. Badminton Aerodynamic Model

Badminton can be regarded as a four-dimensional space. When the shuttlecock leaves the racket and flies in the air, we need to consider the size and height of the shuttlecock and the external factors such as the size and height of the badminton court. We also have to consider a time vector, which makes the technique of playing, the speed of playing, and the ability of human movement [17]. Due to the small size and lightness of the shuttlecock, it is easily affected by various external factors when it is flying in the air. For example, suppose the speed of wind is greater than a certain level. In this case, it will significantly affect its performance under the action of the wind. Moreover, even if the shuttlecock is small and lightweight, it will be affected by the earth's gravitational force. Shuttlecock will also be affected by the air force during the flight and will also be affected by its rotation. The air force is also known as air resistance. It is much more complicated than gravity, and it will change due to factors such as air viscosity. In addition, the shuttlecock will receive a lateral force orthogonal to the speed direction during the flight, causing the shuttlecock to rotate during the flight. Under the action of this force, the shuttlecock's trajectory will deviate from an arc-shaped trajectory. It is the Magnus effect in fluid mechanics [18]. Figures 1(a)–1(c) show the head-on resistance, air friction, and eddy current resistance of the badminton.

The air force on the shuttlecock can be divided into three components in different directions. They are various resistances *X* during the flight of the shuttlecock, the lift *Y* that prevents the shuttlecock from falling vertically due to the influence of gravity, and the departure of the shuttlecock from its original position, the lateral force *Z* of the flight path. It can be known from the data that the air force received by the shuttlecock during flight is not only proportional to the area *S* of the shuttlecock but also proportional to the pressure *Q* of the airflow in the air so that the following relational equations can be obtained:

(1) $$\begin{array}{c} X=B_{x}SQ,\\ Y=B_{y}SQ,\\ Z=B_{z}SQ, \end{array}$$

where *B*_*x*_ is the drag coefficient of various resistances received during the flight of the shuttlecock, *B*_*y*_ is the lift coefficient that prevents the shuttlecock from falling due to gravity, and *B*_*z*_ is the lateral force coefficient that causes the shuttlecock to deviate from the original flight path. *S* represents the contact area between the shuttlecock and the air. Generally, the area of the most significant cross section of the shuttlecock is taken as the contact area between the shuttlecock and the air. Therefore, considering the badminton aerodynamic model will help improve the accuracy of badminton hitting action recognition.

### 2.2. Batting Motion Extraction

When the acceleration sensor collects the athlete's acceleration data, it usually lasts several minutes or even tens of minutes, including many batting actions, forming a long section of long data composed of many discrete points. Therefore, it is necessary to segment and extract each batting action of the athlete to facilitate the subsequent classification and recognition [19]. Window segmentation technology is mainly used to extract batting action. Window segmentation is used to segment the data of feather players' multiple batting to obtain multiple windows with the same or different widths. Each window corresponds to players' single batting action. Window segmentation techniques mainly include sliding window segmentation and event window segmentation [19]. In the proposed work, the sliding window technique is applied.

The data segmentation technology based on the sliding window divides a sampling shot signal into several windows of equal length. The two adjacent windows may overlap or not overlap each other. This paper takes the player's forehand to push several times in continuous confrontation as an example to research the sliding window segmentation technique [20]. The sliding window moves along the time axis through a window of fixed width and extracts the batting action, as shown in Figure 2.

Considering that the data sampling frequency is 200 Hz and the badminton batting action generally does not exceed 0.5 seconds, the window width is set to 100 samples to extract the batting action. The calculation equation of net combined acceleration is as follows:

(2) $$\begin{array}{c} a=\sqrt{a_{x}^{2}+a_{y}^{2}+a_{z}^{2}-1},\\ A_{m}=\arg\underset{m}{\max}\left[\frac{1}{k}\sum_{m}^{m+k-1}a_{m}^{2}\right], \end{array}$$

where *a*_*x*_, *a*_*y*_, *a*_*z*_ is the three-axis acceleration signal and −1 is the always existing gravitational acceleration component, so *a* is the net acceleration representing pure human action, and the unit of acceleration is *g*.

## 3. Methodology

### 3.1. Hidden Markov Model (HMM)

The HMM is a probabilistic model about time series, which describes generating a random series of nonobservable states from a hidden Markov chain and generating an observation from each state to generate a random observation series.  Figure 3 shows the schematic diagram of the proposed HMM [21].

The hidden Markov model is determined by the initial probability distribution *π*, the state probability distribution *A*, and the observation probability distribution *B*. It is defined as follows: let *Q* be the set of all possible states and *V* be the set of all possible observations; then,

(3) $$\begin{array}{c} \left\{\begin{array}{c} Q=\left\{q_{1},q_{2},\ldots ,q_{N}\right\},\\ V=\left\{v_{1},v_{2},\ldots ,v_{M}\right\}, \end{array}\right. \end{array}$$

where *N* is the number of possible states and *M* is the number of possible observations. *I* is the state sequence of length *T*, and *O* is the corresponding observation sequence; then,

(4) $$\begin{array}{c} \left\{\begin{array}{c} I=\left\{i_{1},i_{2},\ldots ,i_{T}\right\},\\ V=\left\{v_{1},v_{2},\ldots ,v_{M}\right\}. \end{array}\right. \end{array}$$

Let *A* be the state transition probability matrix:

(5) $$\begin{array}{c} A={\left[a_{ij}\right]}_{N\times N}. \end{array}$$

Let *B* be the observation probability matrix:

(6) $$\begin{array}{c} B={\left[b_{j}\left(k\right)\right]}_{N\times M}. \end{array}$$

Let *π* be the initial state probability vector:

(7) $$\begin{array}{c} \pi =\left(\pi_{i}\right). \end{array}$$

Therefore, the HMM *λ* can be expressed by the following equation:

(8) $$\begin{array}{c} \lambda =\left(A,B,\pi \right), \end{array}$$

where *A*, *B*, and *π* are called the three elements of the hidden Markov model.

### 3.2. Badminton Action Recognition Based on the Improved HMM

Because of the time sequence of badminton action, it can be modeled by the HMM, which is a probability model about the time sequence. The HMM modeling mainly depends on three parameters: initial probability, transition probability, and observation probability. For each stroke, we establish a set of HMMs applicable to the stroke. Each stroke action is divided into *N* meta-actions with a time sequence. The codebook corresponding to each meta-action is determined through vector quantization, which is the observation set defined by the HMM [16].

The recognition process of badminton action is that the observation sequence of the current hitting action extracted by the preprocessing algorithm [22, 23] is used to input each established HMM of the hitting action. The probability of the optimal state sequence of the current hitting action in each model is obtained using the Viterbi algorithm. The Viterbi algorithm is a dynamic algorithm for obtaining the maximum posterior probability estimate of the most likely sequence of the hidden Viterbi path that results in a sequence of observed events, especially hidden Markov models (HMMs). The hitting action corresponding to the model with the largest probability output is the recognition result of the current observation sequence.

Since multiple datasets aim at the same hitting action in the sample and the sample based on which the training HMM parameter model is based is a single sample, the model data may fall into the local optimum. In contrast, the recognition rate of other samples is low [18]. For multiple training [24, 25], this paper proposes two schemes. One is the mean training method, which integrates the data layer of the input of the model, namely, the observation sequence of the sample, and carries out model training after taking the mean value of multiple groups of training data under the same model. Secondly, the frequency weighted training method is used to linearly weight the frequency of the sample observation sequence in the model and set the sequence of *M* observation values as *O*^(m)^. *M* and *P*_*m*_ are the occurrence frequency of the *m*^th^ observation sequence. Then, the improved calculation equation is as follows:

(9) $$\begin{array}{c} {\bar{\pi }}_{i}=\sum_{m=1}^{M}\frac{\alpha_{1}^{m}\left(i\right)\beta_{1}^{m}\left(i\right)}{P\left(O^{\left(m\right)}|\lambda \right)},\\ {\bar{a}}_{ij}=\frac{\sum_{m=1}^{M}\sum_{t=1}^{T_{m}-1}\alpha_{1}^{\left(m\right)}\left(i\right)a_{ij}b_{j}\left(O_{t+1}^{\left(m\right)}\right)\beta_{t+1}^{\left(m\right)}\left(j\right)}{\sum_{m=1}^{M}P_{m}\sum_{t=1}^{T_{m}}\alpha_{t}^{\left(m\right)}\left(i\right)\beta_{t}^{\left(m\right)}\left(j\right)},\\ {\bar{b}}_{j}\left(k\right)=\frac{\sum_{m=1}^{M}P_{m}\sum_{t=1}^{T_{m}-1}\alpha_{t}^{\left(m\right)}\left(i\right)\beta_{t}^{\left(m\right)}\left(j\right)I\left(o_{t},v_{k}\right)}{\sum_{m=1}^{M}P_{m}\sum_{t=1}^{T_{m}}\alpha_{t}^{\left(m\right)}\left(i\right)\beta_{t}^{\left(m\right)}\left(j\right)}, \end{array}$$

where *α*_t_^(m)^(*i*) and *β*_t_^(m)^(*i*) are the forward probability and backward probability of the *m*^th^ sequence, respectively, and ${\bar{\pi }}_{i}$, ${\bar{a}}_{ij}$, and ${\bar{b}}_{j}\left(k\right)$ are the improved initial, transition, and observation probability parameters, respectively.

The improved HMM training and recognition processes are shown in Figure 4, the training sample data for ten kinds serve as 100 shots of all data, the corresponding model is obtained by the improved training algorithm, and for anyone to identify the strokes, the strokes of the observation are obtained by the data preprocessing algorithm sequence through the Viterbi algorithm. Moreover, 70% of the data was used for training and 30% for testing the HMM. The conditional probability of the occurrence of the optimal state sequence under ten batting action models was calculated, and the model corresponding to the maximum conditional probability was found. The batting action corresponding to the model was the recognition result.

## 4. Experiments and Results

### 4.1. Experimental Setup

This system adopts the MATLAB 2020 development environment and IntelliJ IDEA 2018 (JDK 1.8), the upper computer operating system is Win10, and Bluetooth 4.0 is used for data transmission. The hardware platform of the system is mainly composed of six-axis acceleration sensors. Three of the six sensors are worn by each player. One is attached to the end of the racket handle, and the other two are worn around the player's ankles. The player's hitting signal data [26] collected by the sensor fixed on the end of the badminton racket handle are used for feature extraction of the hitting action. The player's running signal data collected by the sensor fixed on the ankle are used for the restoration and training of the controlled pace.

### 4.2. Feature Extraction of Badminton Hitting Action

Badminton hitting action contains many important characteristics, such as explosive power, hitting speed, and hitting kinetic energy. Therefore, this article compares the important characteristics of badminton players with three different technical levels to quantitatively analyze a single badminton action. A case study, including three different technical levels' player information, is given in Table 1.

As the main scoring point of the hitting action in badminton, the high ball plays a decisive role in the badminton game. The hitting speed, reaction speed, the player's instantaneous explosive power, and the hitting kinetic energy generated during the start and stop of the hit are all important technical characteristic indexes to measure the quality of high-range shots.

### 4.3. Experimental Results

#### 4.3.1. Recognition Performance of the Proposed HMM

The recognition accuracy of the proposed HMM was computed using a confusion matrix. We used the numbers 1–10 to represent 10 different badminton shots, serving, forehand rubbing, and backhand are among the skills you can learn.  Figure 5 shows the confusion matrix of the experimental results in this article.

It can be seen from Figure 5 that the proposed improved HMM has achieved accurate recognition results of 95% in 10 different ball-hitting motion recognition tasks, which proves the effectiveness of the model in this paper.

#### 4.3.2. Comparison with the Traditional HMM

Table 2 provides a comparison between the traditional HMM and the proposed improved HMM. Compared with the traditional HMM, the average recognition rate of the improved HMM is improved by 7.3%. The total recognition rate of the final strokes can reach up to 95% for the proposed improved HMM. Therefore, the proposed model is helpful to improve the competitive level of badminton players.

#### 4.3.3. Effect of Window Length on Recognition Performance

For badminton action recognition, fast response time is desired for real-time applications. In the third study, the nonoverlapped window segmentation scheme was applied to acceleration signals before investigating the impact of window size on the model's performance. Window length created significant effects on classification accuracy. Classification accuracies tended to decrease as window size was increased. The overall classification accuracy dropped from 95% to 90% when the analysis window length was increased from 100 samples to 300 samples, as shown in Table 3. It was observed that a smaller window provided relatively high classification accuracy in badminton action recognition.

#### 4.3.4. Performance Comparison of Different Classification Algorithms

In order to further prove the superiority of the proposed model, we also conducted a comparative experiment with the SVM and BP network. The comparative experimental results are shown in Figure 6.

It can be seen that the model in this paper has a higher recognition rate (more than 90%) than the other two methods (less than 80%). Therefore, this paper adopts the improved HMM method to identify ten different badminton stroke movements. The average recognition rates for the same player can reach 95%, which proves the superiority of the algorithm in this paper.

## 5. Conclusion

This paper proposes an algorithm for badminton hitting action recognition. The system uses a single acceleration sensor fixed at the end of the badminton racket handle to collect the data of the badminton movement. The sliding window data segmentation technique is applied to extract the hitting signal. An improved hidden Markov model is developed to identify ten common badminton shots, serving, forehand rubbing, and backhand are among of the skills you can learn. Experiments show that the algorithm can recognize ten common shots in real time. The average recognition rate of the improved HMM is 7.3% higher than that of traditional HMMs. The final comprehensive recognition rate of shots can reach up to 95%. The model can be used to improve the competitive level of badminton players.

## 6. Limitations and Future Work

The main limitation of this work is that, in the data collection process, only acceleration sensors were used by fifteen sportsmen to recognize ten basic badminton shots. We will plan to extend our approach by including more players and extend the dataset to other sport activities in our future work.

## Figures and Tables

**Figure 1:** Shuttlecock dynamic during flight: (a) the head-on resistance of the badminton, (b) air friction on the badminton, and (c) eddy current resistance on the badminton.

**Figure 2:** Window segmentation technique.

**Figure 3:** Schematic diagram of the hidden Markov model.

**Figure 4:** Improved HMM badminton hitting action recognition model.

**Figure 5:** Confusion matrix of ten badminton shots.

**Figure 6:** Comparison results of different methods.

**Table 1:** Player information of three different skill levels.

Player category	Player description	Number of players
Professional athlete	The second- and third-level badminton players of the Physical Education Institute	5
Amateur	Member of the badminton association	5
Novice	Lab classmates who rarely play badminton	5

**Table 2:** Performance comparison with the traditional HMM.

Classification algorithm	Accuracy (%)
Traditional HMM	87.7
Improved HMM	95

**Table 3:** Performance of different window sizes.

Classification algorithm	Window size (number of samples)	Accuracy (%)
HMM	100	95
	150	93
	200	90

## Data Availability

The data used to support the findings of this study are included within the article.
